The article "Clinical Analysis of Surgical Treatment of Senile Intertrochanteric Fracture Based on Intelligent Knowledge of Health Care" was retracted in 2023. Reasons: signs of a paper mill; suspected computer-generated content; unreliable results or conclusions; lack of ethics approval or compliance.

# Clinical Analysis of Surgical Treatment of Senile Intertrochanteric Fracture Based on Intelligent Knowledge of Health Care

**DOI:** 10.1155/2022/3556330

**Published:** 2022-07-06

**Authors:** Weidong Bi, Jianjie Xu, Zhihui Dong, Zhaona Wang, Jiebing Li, Yongwei Shang, Jianzhong Wu

**Affiliations:** The Second Department of Orthopedics, Shijiazhuang People's Hospital, Shijiazhuang 050000, China

## Abstract

In order to explore the clinical application value of intelligent health care knowledge combined with closed reduction intramedullary nail fixation in elderly patients with intertrochanteric fracture of the femur, a retrospective analysis is performed on 80 elderly patients who received intertrochanteric surgery from January 2019 to January 2021. All patients were divided into study group and control group based on intelligent medical knowledge received or not. During the phase of treatment, both the two groups were treated with closed reduction and intramedullary nailing. The control group received conventional knowledge training and rehabilitation before and after the surgery, and the research group received additional intelligent medical knowledge health care. Observations of patients after bed and ground time are compared and the VAS score is used to evaluate the pain degree at 12 h, 24 h, and 48 h after surgery. Besides, the incidence of postoperative complications in the two groups is observed. From the clinical follow-up results, it is clearly evident that intramedullary nail fixation based on medical care knowledge can effectively improve the hip function and quality of life in patients, reduce postoperative pain, and improve the prognosis of elderly patients with femoral trochanteric fracture.

## 1. Introduction

Intertrochanteric fracture of femur refers to the fracture from the base of femoral neck to the level above the lesser trochanter. It is also a common injury in the elderly patients. Due to the abundant blood circulation in the trochanter, there is little non-union after the fracture. Intertrochanteric fracture of femur usually occurs in the elderly patients. This is because most elderly people have osteoporosis, which is likely to cause fractures in this part. The typical manifestation is hip pain and unable to stand and walk normally. The specific type of intertrochanteric fracture can be judged by local X-ray, CT, and three-dimensional reconstruction. According to the statistical results, intertrochanteric fractures account for 7.01% of adult systemic fractures; and the elderly over 65 years old account for 23.79% of systemic fractures [1]. At present, intertrochanteric fracture of the femur is treated with surgical fixation, and conservative treatment has a high incidence of complications. As China gradually enters an aging society, only 30% of patients can recover to a life before the injury. Many people die of complications without effective treatment. The disease brings high mortality, nonunion, and teratogenesis rates, and high treatment costs. Some experts estimate that by 2020, the medical cost of hip fractures in China will reach 60 billion US dollars. The increase in medical burden and poor prognosis leads to the decline of patients' quality of life, which brings a heavy economic burden to patients' families, and society [2, 3]. For the elderly patients with femoral intertrochanteric fracture, the clinical treatment includes conservative treatment and surgical treatment. Conservative treatment is mainly long-term bed traction, which usually leads to systemic complications. Within 2 weeks after the trauma, due to the decline of immune function, the incidence rate of pneumonia and infectious diseases is high. In addition, there are many surgical treatments, such as dynamic hip internal fixation, closed reduction and intramedullary nail fixation, and artificial hip replacement. However, there are still some disputes on the choice of the surgical scheme [4, 5]. In addition, some studies have also pointed out that due to the lack of medical care knowledge of elderly patients, they choose to stay in bed for a long time, so as not to affect their postoperative recovery, which is easy to cause muscle atrophy and joint stiffness. Therefore, popularizing medical care knowledge is also of great significance to such patients [6]. The aging of the population will directly lead to the rapid growth of the medical and health care needs of the elderly and form greater pressure on social medical resources [7]. In addition to continuing research on medical technology, people have found that the rational use of the empowerment from digital technology is likely to be the “golden key” to solve the problem [8]. Smart medicine has significant advantages in home medical services, remote consultation, and remote medical education services. Therefore, in this study, 80 elderly patients admitted to our hospital for intertrochanteric fracture from January 2019 to January 2021 were treated with closed reduction intramedullary nailing combined with intelligent healthcare knowledge to observe its impact on the prognosis of these patients.

This paper is organized as follows. In Section 2, the related work is reviewed. In Section 3, we present the general information and proposed method. In Section 4, the experimental results and analysis is discussed. Finally in Section 5, some concluding remarks are made.

## 2. Related Work

Intertrochanteric fracture of femur is a common injury in the elderly. Since most of the elderly are accompanied by chronic diseases such as hypertension and hyperglycemia, many nonsurgical complications are prone to occur in clinical treatment and lead to poor prognosis. Conservative treatment will further lead to bone nonunion and malunion in elderly patients. Long-term bed rest will also lead to muscle atrophy, joint stiffness, and pressure sores. These problems seriously threaten the physical and mental health of the elderly patients. Therefore, appropriate medical care knowledge and effective surgical treatment are of great significance to the prognosis of elderly patients with a femoral intertrochanteric fracture [9]. In current clinical according to a rotor between femur fractures have a variety of surgical plans, including the intramedullary nail fixation, and artificial hip replacement, can to a certain extent, improve the effect of fracture healing, recovery of hip joint function, and improve patients but treatment above is pure treatment, has yet to see the combined surgery and wisdom medical care and comparing observation curative effect [10]. Based on this, this study used medical care knowledge to carry out rehabilitation training for elderly patients with an intertrochanteric fracture on the basis of intramedullary nail fixation and analyzed its application value for elderly patients with intertrochanteric fracture.

In preoperative elderly patients in advance in order to explain the procedure and to reduce the patients' fear of surgery, the postoperative activity can therefore be carried out in the field of rehabilitation training. This study shows that the bed activity time and bed activity time of the team are shorter than those of the control group. And it can also illustrate the above views; preoperative intelligent health care knowledge can reduce the psychological burden of patients. It can help patients get out of bed early and move around and shorten the bed time [11]. In addition, there were no significant difference in postoperative complications between the two groups, but the infection rate of the study group was slightly lower than that of the control group; hence, in this analysis, the authors' speculation may be due to two groups of patients who use surgery the same way, so the postoperative complications contrast will not have a too big difference, but the team in preoperative intelligent health care knowledge training, compared with the control group, have a more detailed understanding of what behaviors may cause infection by pulling the wound after surgery, so they pay more attention to these aspects, resulting in a lower wound infection rate [12]. At the same time, in postoperative patients with lower limb venous thrombosis. causes are due to the fact that elderly are more worried about postoperative activities, no effective exercise lower limbs resulted in part of patients with lower extremity venous thrombosis, but the team received preoperative intelligent health care knowledge training. They have higher compliance and consciousness to postoperative rehabilitation treatment, as well as higher awareness of self-management, so the incidence of venous thrombosis of lower limbs is slightly lower [13]. As this study is to evaluate by the Harris Hip Function, the results show two groups of patients with postoperative hip joint function improved, though six months after hip function had no significant difference in both the groups, but the study group 1 month after the surgery of the hip joint function was significantly better than control group, analyzes reasons for this recognition on the above as soon as possible after the activity and the benefits of exercise are fully understood. Therefore, in the short term after surgery, patients can actively cooperate with rehabilitation exercise, so that patients can improve the function of hip joint earlier [14–17]. In addition two kinds of treatment not only can improve the elderly patients with femoral fractures between rotor hip function, also can effectively improve the quality of life, and the team 1 months and 6 months after surgery improved quality of life of significantly higher, illustrate the team earlier recovery of hip function in patients with better blend in social activities, the ability to live independently, Therefore, the quality of life is higher [18, 19].

## 3. General Information and Proposed Methods

### 3.1. General Information

A retrospective analysis was performed on 80 elderly patients who underwent intertrochanteric surgery in our hospital from January 2019 to January 2021, and they were randomly divided into study group (*n* = 40) and control group (*n* = 40). The study group included 22 female patients and 18 male patients, aged 61–78 years. The average age was (67.43 ± 7.42) years. There were 20 female and 20 male patients in the control group, aged from 60 to 78 years old, with an average of (67.03 ± 7.39) years old. There were no significant difference in the baseline data between the two groups (*P* > 0.05), which was comparable. All patients enrolled in the study signed informed consent before the surgery and obtained the right to know the contents of intraoperative procedures and postoperative follow-ups.

Inclusion criteria are as follows [20]: (1) meet the clinical diagnostic criteria for intertrochanteric fracture of femur; (2) complete clinical imaging diagnostic data and general information; (3) the treatment compliance is high and can cooperate with the study; (4) Good communication and understanding skills.

Exclusion criteria are as follows [21]: (1) accompanied by mental diseases, unable to communicate with researchers normally; (2) lost contact or quit during the follow-up period; (3) the body cannot tolerate the operation; (4) poor treatment compliance cannot be coordinated with the study.

### 3.2. Methods

#### 3.2.1. Surgical Methods

Both the groups were treated with closed reduction and intramedullary nail fixation during the operation. The specific operation steps are as follows: (1) during the operation, the patients were in lateral or supine position and were anesthetized with general anesthesia and nerve block with an auxiliary line; (2) after the anesthesia took effect, fracture reduction and traction were performed first; (3) make a 5 cm incision upward at the top of the greater tubercle of femur, open the piriform fossa along the muscle fibers of the median longitudinal incision, and slowly move the needle with the greater trochanter area as the midpoint; (4) the medullary cavity was expanded with a bone marrow expander until there was a suitable surgical space; (5) then continue to push the intramedullary nail and fix it with the nail tail cap; (6) the wound was rinsed with normal saline, a drainage tube was left and sutured layer by layer.

Finally, both the groups were treated with broad-spectrum antibiotics for 24 hours to prevent infection.

#### 3.2.2. Popularization of Intelligent Healthcare Knowledge

In the control group, the relevant knowledge of postoperative rehabilitation and health care was popularized to the patients before the surgery, and the patients were instructed to carry out corresponding rehabilitation training after the surgery to promote the recovery of body functions. The specific contents included: (1) ankle dorsiflexion and quadriceps muscle training, through the maximum flexion and extension of the ankle joint and resistance training according to the patient's personal situation, hip flexion and knee bend 30°–40° training; (2) three days after the surgery, the affected limb coasting rehabilitation was started, and the hip flexion and knee bend Angle were increased to 40°–60°; (3) five days after the surgery, walking training should be conducted with the assistance of medical staff or family members according to the patient's recovery. If pain or physical intolerance occurs during this training, the training should be stopped immediately; (4) voluntary hip movement can be performed about 4 weeks after the surgery, but the hip flexion and knee bend Angle should not exceed 90°, and weight training should not be avoided.

Compared with the control group, the research group received additional intelligent medical knowledge health care. The specific contents include: (1) preoperative video interpretation about the operation process of the related content, popularize knowledge related to the operation, reduce the psychological burden of patients for surgery, so as to help patients keep relaxed, good response to treatment, and improve the follow-up rehabilitation compliance; (2) arrange professional rehabilitation personnel to simulate correct postures for patients before surgery, and explain how to protect themselves with correct postures in case of emergencies such as falls; (3) explain the possible causes of postoperative pain aggravation, and teach patients how to take effective measures to relieve the pain. If the pain is unbearable, they can seek doctors to use appropriate analgesic drugs.  Figure 1 illustrates the technical route.

#### 3.2.3. Harris Hip Function Score

The scale was mainly used to evaluate the effect of hip replacement, including pain degree, daily functional performance, and range of motion, among which pain degree was scored 44 points, daily functional performance was scored 51 points, and range of motion was scored 5 points. The score range of this scale is 0 to 100, and the lower the score is, the worse the hip joint function is, unable to independently complete daily living operations.

#### 3.2.4. World Health Organization Quality of Life (WHOQOL)

This scale has altogether four areas, respectively from the life health, feeling of things, action ability and the negative emotions seizure frequency was carried out on the quality of life assessment, and the top three areas respectively according to very poor, poor, in general, good, very good for 1 ∼ 5 points, respectively, according to the fourth field never, rarely, sometimes, often, always remember to 5 ∼ 1 points. The scale ranges from 0 to 100, with a higher score indicating a better quality of life.

#### 3.2.5. Visual Analogue Scale (VAS)

This scale is mainly used to evaluate the pain degree of patients. The specific operation is to draw a line with a length of 10 cm on the paper, with one end marked as 0, indicating no pain. The other end is marked with a 10, indicating extreme pain, and patients are asked to mark on a straight line according to their own perception of pain. Scores ≤3 indicate mild pain and tolerable; A score of 4–6 indicates that the pain has affected sleep but is still tolerable. A score of ≥7 indicates pain that is unbearable and interferes with daily life.

### 3.3. Observation Indicators

The observation indicators include: (1) observe the postoperative time in bed and on the ground; (2) VAS score was used to compare the pain degree at 12h, 24h, and 48h after surgery; (3) the incidence of postoperative complications in the two groups was observed; (4) Harris Hip Function score was used to evaluate the hip function of the two groups before surgery, 1 month and 6 months after surgery; (5) the changes of quality of life in the two groups before and after treatment were compared.

### 3.4. Statistical Processing

SPSS 25.0 statistical software was used for data analysis. (1) Measurement data: a normality test was performed on the data first. If the data followed normal distribution and homogeneity of variance, it was represented by mean ± standard deviation. Paired sample *t* was used for testing within the group, and variance comparison was used between groups. Repeated measurement anOVA was used between multiple groups to conduct spherical test. (2) Count data: descriptive statistical analysis was conducted by percentage, and *x*^*2*^ test was performed. *P* < 0.05 indicates significant difference.

## 4. Experimental Results and Analysis

### 4.1. Comparison of Intraoperative Blood Loss, Operation Time, and Postoperative Time in Bed and on the Ground

Compared with the control group, the bed time and ground time of the study group were significantly shortened (*P* < 0.05), as shown in Table 1.

### 4.2. VAS Score Was Used to Evaluate the Pain Degree at 6 h, 12 h, and 24 h after Surgery

Postoperative pain in both groups decreased, and pain in the study group at 12 and 24 hours postpartum was significantly lower than that of the control group (both *P* < 0.05), as shown in Table 2. The symbol “^*∗*^” indicates that compared with 6h after surgery, *∗P* < 0.05; “#” indicates that compared with 12h after surgery, #*P* < 0.05. In Figure 1, “a, b, c” indicates that if the same letter is shared, *P* > 0.05; if no common letter is shared, *P* < 0.05. Besides, the symbol “#” means the comparison of two components at the same time point *P* < 0.05.

Figure 2 is the differences in pain at different time points between the two groups.  Figure 3 shows the volcanic map of difference between two groups at time points.

### 4.3. Incidence of Postoperative Complications

There was no significant difference in the incidence of total complications between the two groups, but the incidence of postoperative venous thrombosis and hip varus in the control group was slightly higher than that in the study group, as shown in Table 3.

### 4.4. Hip Function Evaluation

After treatment, the hip function increased in both groups, and there was a significant difference in hip function between the two groups 1 month after surgery (*P* < 0.05), and no difference was observed in other time periods, as shown in Table 4 and Figures 4 and 5. The symbol “^*∗*^” indicates that compared with preoperative, ^*∗*^*P* < 0.05; “#” indicates that compared with 1 month after surgery, ^#^*P* < 0.05. In Figure 4, “a, b, c” means that if the same letter is used, there is no significant difference between time points; “#” means that there is a significant difference between the two groups at the same time point.

### 4.5. Quality of Life Evaluation

Compared with before treatment, the quality of life in both groups improved after treatment, and the quality of life in the study group was significantly higher than the control group at 1 and 6 months after surgery (*P* < 0.05), as shown in Table 5 and Figure 6. The symbol “^*∗*^” indicates that compared with preoperative, ^*∗*^*P* < 0.05; “#” indicates that compared with 1 month after surgery, ^#^*P* < 0.05. In Figure 6, “a, b, c” means that if the same letter is used, there is no significant difference between time points; “#” means that there is a significant difference between the two groups at the same time point.

## 5. Conclusion

In this study, clinical analysis of the surgical treatment of a senile intertrochanteric fracture based on intelligent knowledge health care is conducted. From the clinical follow-up results, it is clearly evident that intramedullary nailing based on intelligent medical knowledge can effectively improve the hip function and quality of life of patients, and can help patients with early walking training. Moreover, it can improve the speed of hip recovery, which plays an important role in improving the prognosis and quality of life of patients.

## Figures and Tables

**Figure 1:** Technology roadmap.

**Figure 2:** Differences in pain at different time points between the two groups.

**Figure 3:** Volcanic map of difference between two groups at time points.

**Figure 4:** Trends of hip function in the two groups.

**Figure 5:** Preoperative and postoperative X-ray images: (a) the preoperative indication of left intertrochanteric fracture of the femur; (b) good reduction of fracture site after operation; (c) be fixed and stable 3 months after surgery, and the fracture site began to heal; (d) the healing of fracture site and no loosening of internal fixation 6 months after surgery.

**Figure 6:** Trends of quality of life in the two groups.

**Table 1:** Comparison of intraoperative and postoperative indicators.

Group	Number	Bed time (d)	Ground walking time (d)
Study group	40	2.17 ± 0.64	5.62 ± 1.25
Control group	40	3.04 ± 0.73	6.83 ± 1.72
*t*		5.668	3.559
*P*		＜0.001	0.001

**Table 2:** Comparison of pain degree at 6 h, 12 h, and 24 h after surgery.

	Number	6 h	12 h	24 h	*F*	*P*
Control group	40	7.27 ± 1.28	5.21 ± 1.23^*∗*^	4.37 ± 1.22^∗#^	4.2723	＜0.001
Study group	40	7.25 ± 1.26	4.58 ± 1.18^*∗*^	3.75 ± 1.04^∗#^	4.284	＜0.001
*t*		0.089	2.943	8.009		
*P*		0.929	0.017	＜0.001		

**Table 3:** Comparison of complications.

Group	Number	Vein thrombosis	Infection	Hip varus	Total complications
Study group	40	1 (2.50%)	1 (2.50%)	1 (2.50%)	3 (7.50%)
Control group	40	4 (10.00%)	3 (7.50%)	2 (5.00%)	9 (22.50%)
*x* ^*2*^					3.529
*P*					0.060

**Table 4:** Hip function evaluation.

Group	Number	Preoperative	1 month after surgery	6 month after surgery	*F*	*P*
Study group	40	46.63 ± 6.43	59.42 ± 7.42^*∗*^	74.34 ± 10.23^∗#^	9.524	＜0.001
Control group	40	45.33 ± 6.29	54.54 ± 6.68^*∗*^	72.73 ± 10.04^∗#^	9.043	＜0.001
*t*		0.914	3.091	0.710		
*P*		0.364	0.003	0.480		

**Table 5:** Quality of life evaluation.

Group	Number	Preoperative	1 month after surgery	6 month after surgery	*F*	*P*
Study group	40	51.23 ± 9.53	67.43 ± 12.23^*∗*^	79.43 ± 13.41^∗#^	8.324	＜0.001
Control group	40	50.23 ± 9.84	60.32 ± 11.29^*∗*^	71.22 ± 12.24^∗#^	7.394	＜0.001
*t*		0.462	2.702	2.860		
*P*		0.646	0.008	0.005		

## Data Availability

The simulation experiment data used to support the findings of this study are available from the corresponding author upon request.
